# Intelligent Energy-Aware Thermal Exchange Optimization with Deep Learning Model for IoT-Enabled Smart Healthcare

**DOI:** 10.1155/2023/3830857

**Published:** 2023-07-14

**Authors:** Mahmoud Ragab, Sami Saeed Binyamin

**Affiliations:** ^1^Information Technology Department, Faculty of Computing and Information Technology, King Abdulaziz University, Jeddah 21589, Saudi Arabia; ^2^Department, Faculty of Science, Al-Azhar University, Nasr City 11884, Cairo, Egypt; ^3^Centre for Artificial Intelligence in Precision Medicines, King Abdulaziz University, Jeddah 21589, Saudi Arabia; ^4^Computer and Information Technology Department, The Applied College, King Abdulaziz University, Jeddah 21589, Saudi Arabia

## Abstract

In recent years, Internet of Things (IoT) and advanced sensor technologies have gained considerable interest in linking different medical devices, patients, and healthcare professionals to improve the quality of medical services in a cost-effective manner. The evolution of the smart healthcare sector has considerably enhanced patient safety, accessibility, and operational competence while minimizing the costs incurred in healthcare services. In this background, the current study develops intelligent energy-aware thermal exchange optimization with deep learning (IEA-TEODL) model for IoT-enabled smart healthcare. The aim of the proposed IEA-TOEDL technique is to group the IoT devices into clusters and make decisions in the smart healthcare sector. The proposed IEA-TEODL technique constructs clusters using the energy-aware chaotic thermal exchange optimization-based clustering (EACTEO-C) scheme. In addition, the disease diagnosis model also intends to classify the collected healthcare data as either presence or absence of the disease. To accomplish this, the proposed IEA-TODL technique involves several subprocesses such as preprocessing, K-medoid clustering-based outlier removal, multihead attention bidirectional long short-term memory (MHA-BLSTM), and weighted salp swarm algorithm (WSSA). The utilization of outlier removal and WSSA-based hyperparameter tuning process assist in achieving enhanced classification outcomes. In order to demonstrate the enhanced outcomes of the IEA-TEODL approach, a wide range of simulations was conducted against benchmark datasets. The simulation results inferred the enhanced outcomes of the IEA-TEODL technique over recent techniques under distinct evaluation metrics.

## 1. Introduction

With the advancements made in smart sensorial media, Internet of Things (IoT), and cloud techniques, smart health care has gained considerable interest in different domains such as healthcare, academia, government, and industry [1]. In recent times, Internet of Things (IoT) has brought the vision of a smart world into reality, with numerous services in the pipeline generating massive amounts of data. Cloud computing (CC) suits well as an enabling technique since it presents a flexible stack of software, computing, and storage services at a lower cost [2]. Cloud-based service has the potential to provide a high-quality seamless experience to clinicians, physicians, and other caregivers, anytime and anywhere. While research has been making advances in cloud services and IoT separately, minimum attention has been paid to emerging, affordable, and cost-effective intelligent healthcare services [3]. At present, cloud and IoT technologies have assisted in delivering smart healthcare services on a real-time basis and also have made considerable improvements.

With the integration of the IoT cloud, a great demand for intelligent and smart healthcare systems provides a rapid and seamless response. Artificial intelligence (AI) and deep learning (DL) techniques can improve decision-making and cognitive behaviour [4]. Advanced electronic applications are presented to intelligent healthcare stakeholders along with smart sensor devices. In spite of these, it is challenging to access or find hospitals and medical professionals in intelligent healthcare environments. In general, patients with serious medical needs must be provided quick attention and faster response in order to save their lives [5]. Therefore, data recorded from patients needs to be interpreted and transferred to healthcare professionals with minimum delay while the results need to be sufficiently accurate so that it can be utilized by healthcare experts for disease prognosis. Hence, a smart healthcare system is required that could resolve the above-mentioned problems and leverage the technology and services available in the intelligent healthcare environment.  Figure 1 illustrates the structure of a smart healthcare system.

Though there have been advancements in this domain, the concept of a smart healthcare system remained uncertain without cognitive function. Smart city service can never be exploited completely without the cognitive knowledge of its stakeholders [6]. Even though the conventional methods achieve rapid delivery of results, it is expected to obtain highly accurate results. But, most of the time, the results suffer from complex data [7]. In this situation, high accuracy can be accomplished by deep learning (DL) techniques and its different versions. In literature, these techniques are trained using large datasets [8]. DL method is an emerging field that has gained considerable outcomes in sequence prediction, mixed-modality data sets, and natural language processing tasks that have received heavy growth in various applications such as computer vision and speech recognition [9, 10].

The current article develops intelligent energy-aware thermal exchange optimization with deep learning (IEA-TEODL) model for IoT-enabled smart healthcare. The proposed IEA-TEODL technique derives energy-aware chaotic thermal exchange optimization-based clustering (EACTEO-C) scheme. Besides, a disease diagnosis model is also involved to classify the collected healthcare data into either presence or absence of the disease. To accomplish this, the proposed IEA-TODL technique involves several subprocesses such as preprocessing, K-medoid clustering-based outlier removal, multihead attention bidirectional long short-term memory (MHA-BLSTM), and weighted salp swarm algorithm (WSSA). In order to validate the promising performance of the IEA-TEODL technique, a wide range of simulations was performed against benchmark datasets, and the results were validated under different measures.

## 2. Literature Review

Mansour et al. [11] developed a disease diagnosis system for diabetes and heart disease using IoT and AI convergence methods. The presented technique employed crow search optimization approach-based cascaded LSTM (CSO-CLSTM) for disease diagnoses. To accomplish improved classification of healthcare information, CSO was employed for tuning “weights” and “bias” parameters of the presented approach. The authors in the literature [12] developed a cloud-centric IoT-based *m*-healthcare monitoring disease diagnosis system that predicts the possible disease occurrence with the severity level. In this study, key terminology was determined to generate user-based health measurement by examining computation science concepts.

In literature [13–15], the authors presented a disease diagnosis system with DL as well as IoT. The healthcare information is preprocessed since it contains noise. The preprocessed information is then passed onto isolation forest (iForest) for outlier recognition with high precision and linear time complexity. The data undergo a classification method in which DenseNet169 and PSO methods are incorporated to diagnose the disease; the parameter is then tuned to improve the performance. Awotunde et al. [16] developed an IoT-WBN-based architecture with an ML approach. The data collected from wearable sensors such as glucose sensors, body temperature, chest, and heartbeat sensors are transferred by IoT device to the cloud dataset.

Nagarajan et al. [17] designed an IoT-based FoG-enabled cloud network framework that accumulates real-time healthcare information from patients through a number of healthcare IoT sensor networks. This information is examined by the DL technique deployed in a fog-based healthcare environment. Moreover, the presented approach was utilized in sustainable smart city solutions to estimate real-time process. Ihnaini et al. [18] proposed an intelligent healthcare system for diabetes based on deep ML and data fusion perspectives. With data fusion, the unrelated burden of computation abilities was removed, and the presented system's efficiency in terms of recommendation and prediction of this severe disease, in a precise format, was increased. At last, the ensemble ML approach was trained for predicting diabetes.

## 3. The Proposed Model

In this study, a novel IEA-TEODL technique has been developed to accomplish clustering and decision-making in an IoT-enabled smart healthcare environment. The proposed IEA-TEODL technique follows 2-stage processes, namely EACTEO-C-based cluster construction and optimal DL-based disease classification. The detailed working process of these two modules is elaborated in the succeeding subsections.  Figure 2 displays the block diagram of the IEA-TEODL technique.

### 3.1. Process Involved in EACTEO-C Technique

In the primary stage, the IoT devices are placed in the healthcare environment to gather medical data from the patients. In order to achieve effectual energy utilization and data transmission to the cloud server, the EACTEO-C technique is executed to select the cluster head (CH) and construct it.

#### 3.1.1. Overview of CTEO Algorithm

The primary aim behind the adaption of a meta-heuristic approach named thermal exchange optimization (TEO) is to cluster the nodes. The model of temperature from TEO reflects the interface feature of nodes [19]. The cooling object mentions the place of nodes whereas the environmental temperature signifies the adjacent nodes. The object is considered as a sensor node. Therefore, important nodes are either interpreted as objects or conversely.

The primary temperature of every node is defined as follows:

(1) $$\begin{array}{c} T_{i}^{0}=T_{\min}+rndx\left(T_{\max}-T_{\min}\right)\text{,} \end{array}$$

where *T*_*i*_^0^ refers to the primary solution vector of the node, *i*. *T*_min_ and *T*_max_ signify the limits of temperature variables. In addition, rnd stands for arbitrary vector, whereas all the components are in the range of zero and one. The main function computes the cost value of all the nodes. The memory has regarded that hierarchy holds the optimum *T* vector, and the main function value is connected to these vectors. It improves the technical performance with no increase in computational cost. In this way, a thermal memory (TM) is utilized to save several optimum solutions at the moment. So, during this phase, solution vectors, stored from TM, are transmitted to populations. In addition, a similar amount of accessible worse nodes is not assumed. Eventually, the node is sorted in an ascending order based on its respective main function values. The node is divided into two equivalent groups. For instance, *T*_1_ is an environment object for *T*_*n*/2+1_ cooling object and conversely.

Generally, if the *β* value of object is lesser, it somewhat modifies the temperatures. An analogy is simulated as this feature is projected. The value of all the nodes is calculated based on equation (2). Therefore, the *β* value of lesser cost node remains a minimum value, and somewhat it modifies the node place.

(2) $$\begin{array}{c} \beta =\frac{cost\left(node\right)}{cost\left(wnode\right)}\text{.} \end{array}$$

The time is dependent upon the number of iterations. *t* denotes the time value for all the nodes and is computed as follows:

(3) $$\begin{array}{c} t=\frac{N_{iter}}{N_{\max\;-iter}}\text{,} \end{array}$$

where *N*_iter_ and *N*_max−iter_ demonstrate the present and maximal number of iterations correspondingly. The environment temperature is replaced by equation (4). At this point, *c*_1_ and *c*_2_ denote control variables.

(4) $$\begin{array}{c} T_{i}^{env}=\left(1-\left(c_{1}+c_{2}*\left(1-t\right)\right)*rnd\right)*T_{i}^{p-env}\text{.} \end{array}$$

*T*_*i*_^*p*−enν^ refers to the previous temperature of the node modified to *T*_*i*_^enν^.

- (1 − *t*) is recognized to decrease arbitrariness when approaching the final iteration. While the procedure is nearing the end, *t* improves and reduces the production of arbitrariness in a linear fashion.
- *c*_1_ checks the size of arbitrary steps. Besides, *c*_1_ contains arbitrariness if it does not utilize a descending method (*c*_2_=0).
- *c*_2_ controls (1 − *t*). That is, where a decrease is not needed, this could be regarded as equivalent to zero.

Where the condition of *C*=0(*c*_1_=*c*_2_=0), the preceding temperature is multiplied by *I*^″^ and *c*_1_ and *c*_2_ are chosen in {0 or 1}. With the preceding stages and equation (4), the upgrade temperature of all the nodes is defined based on equation.

(5) $$\begin{array}{c} T_{i}^{new}=T_{i}^{env}+\left(T_{i}^{prev}-T_{i}^{env}\right)\exp\;\left(-\beta t\right)\text{.} \end{array}$$

*P*_*r*_ parameter from (0,1) defines whether the element of all the nodes is replaced. To all the nodes, *P*_*r*_ is related to rnd(*i*)(*i*=1,2, ⋯, *n*) and is an arbitrary number that is equally distributed from zero and one. If rnd(*i*) < *P*_*r*_, a dimension nodes, *i* is arbitrarily selected, and their values are redefined as follows:

(6) $$\begin{array}{c} T_{ij}=T_{j,\min}+rndx\left(T_{j,\max}-T_{j,\min}\right)\text{,} \end{array}$$

where *T*_*i*,*j*_ refers to the variable *j* of node *i*. *T*_*j*,min_ and *T*_*j*,max_ imply lower as well as upper limits of the variable *j* correspondingly. Only one size is altered to preserve the infrastructure of nodes. This method presents many benefits to nodes for moving throughout the searching region and attaining the optimum diversity.

In this work, the TEO algorithm can be improved with the design of the CTEO algorithm using chaotic concepts [20]. A chaos map employs chaotic variables with changeable nature before arbitrary variables. This order is initiated from nonlinear and dynamic systems whereas nonconvergent orders are from nonperiodic and bounded systems. It can offer easy searching together with a superior convergence rate than arbitrary search. This process uses the technique for providing the optimum exploration from solution spaces due to their dynamic performance of turbulence sequence. The current analysis utilizes a sinusoidal chaotic map function to improve both convergence speed and premature convergence of the TEO technique so as to consider a trade‐off between exploitation as well as exploration techniques. This is performed to provide a well-defined outcome from the solution space which does not stuck at the local optimum points. In order to modify the TEO approach with the help of a chaos map, the chaos value is replaced with arbitrary numbers using the important formula as follows:

(7) $$\begin{array}{c} r_{i+1}=P.r_{i}^{2}\sin\;\left(\pi .r_{i}\right)\text{,} \end{array}$$

where *P* defines the control parameter, and *r*_*i*_ and *r*_*i*+1_ imply the chaotic arbitrary numbers generated from preceding and the existing iterations correspondingly. At this point, *r*_0_=0.7 and *P*=2.3.

#### 3.1.2. Application of EACTEO-C Technique for CH Selection

The primary goal of the EACTCO-C technique is to minimize the distance among the carefully chosen CH nodes. The main objective is to minimize the delay during the transmission of information from one node to another. In contrast, for the network energy should be higher, it should consume a small number of energies at the time of data communication. The objective function of the adapted CH is given in equation (7), where the value of *η* must depend upon 0 < *η* < 1. Now, *v*_*m*_ and *v*_*n*_ show the operations as given as follows. The constraints on distance, delay, and energy are stated as *σ*_1_, *σ*_2_, and *σ*_3_. The condition of this constraint is represented by *σ*_1_+*σ*_2_+*σ*_3_=1. *X*^*x*^ − *B*_*s*_ represents the distance between normal and sink nodes.

(8) $$\begin{array}{c} H_{n}=\eta v_{n}+\left(1-\eta \right)v_{m}\text{,} \end{array}$$

(9) $$\begin{array}{c} v_{m}=\sigma_{1}*v_{i^{dis}}+\sigma_{2}*v_{i^{ene}}+\sigma_{3}*v_{i^{del}}\text{,} \end{array}$$

where *v*_(*m*)_^dis^ represents the packet transmission from the normal node to CH and from CH to BS. *v*_*i*^dis^_ must depend upon [0,1]. The value of *v*_*i*^dis^_ remains high when the normal node is more along with distance among CH [21].

(10) $$\begin{array}{c} v_{i^{dis}}=\frac{v_{\left(m\right)}^{dis}}{v_{\left(n\right)}^{dis}}\text{,}\\ v_{\left(m\right)}^{dis}=\overset{N_{x}}{\underset{x=1}{\sum }}\left[\left\|C_{x}-B_{s}\right\|\right.+\overset{N_{y}}{\underset{y=1}{\sum }}\left\|C_{x}-X_{x}\right\|\text{,}\\ v_{\left(n\right)}^{dis}=\overset{N_{\chi }}{\underset{x=1}{\sum }}\overset{N_{y}}{\underset{y=1}{\sum }}\left\|X_{x}-X_{y}\right\|\text{.} \end{array}$$

*X*_*x*_ denotes the normal node in *x*^th^ cluster, *C*_*x*_ represents the CH of *x*^th^ cluster, the distance between the BS and CH is shown as *C*_*x*_ − *B*_*s*_, *C*_*x*_ − *X*_*x*_ represents the distance between normal node and CH, and *X*_*x*_ − *X*_*y*_ shows the distance among two normal nodes, *N*_*x*_ and *N*_*y*_ indicate the node amount that does not assume *x*^th^ and *y*^th^ cluster. The value of *v*_*i*^ene^_ becomes higher than one, and the whole CH cumulative *v*_(*m*)_^ene^ and *v*_(*n*)_^ene^ is considered as less energy value with high number of CH s.

(11) $$\begin{array}{c} v_{i}^{ene}=\frac{v_{\left(m\right)}^{ene}}{v_{\left(n\right)}^{ene}}\text{.} \end{array}$$

Delta fitness function is directly proportionate to each node that resides in the cluster. Thus, a delay gets reduced, when the CH owns a lesser number of nodes. The denominator *N*_*N*_ shows the overall number of nodes in WSN, and the numerator indicates the high amount of CH. Furthermore, the value of *v*_*i*_^de l^ must be in *d*[0,1].

(12) $$\begin{array}{c} v_{i}^{del}=\frac{\max{\left(\left\|C_{x}-X_{x}\right\|\right)}_{x=1}^{N_{c}}}{N_{N}}\text{.} \end{array}$$

### 3.2. Disease Diagnosis Module

In this work, the disease diagnosis model encompasses a series of subprocesses, namely preprocessing outlier removal, MHA-BLSTM-based classification, and WSSA-based hyperparameter optimization.

#### 3.2.1. Data Preprocessing

At the initial stage, preprocessing takes place in different ways, namely data normalization, data transformation, and data augmentation. In this work, min-max normalization approach is used to normalize the input medical data. Besides, data are also transformed into a useful format, and data augmentation is applied using SMOTE technique to increase the size of the dataset.

#### 3.2.2. K-Medoid Clustering

Next to data preprocessing, the outlier removal process is carried out using the K-medoid clustering approach. The K-means approach that utilizes and determines the means of data point in the calculation is mainly sensitive to the outlier. To resolve this, a new approach was developed in which the medoids are utilized rather than the average value from the cluster. Medoids are centre points from the cluster, and the approach is named as k-medoids clustering. Even though k-medoids computationally increase their demands, the k-medoids cluster is not mainly sensitive to the existence of outlier points and is appropriate to discrete and continuous fields of information [22]. Generally, the input provided has the value of *k* that denotes the amount of clusters determined to data. For every *k* cluster, a *k*-reference point is chosen. The variance between k-medoids and *k*-means algorithms is that the former k-medoids considers the point as a reference object for the cluster whereas *k*-means considers the average value from the former k-medoid cluster as the reference point.

#### 3.2.3. Data Classification Using MHA-BLSTM Model

During the data classification process, the MHA-BLSTM model can be employed for the classification process. RNN is a well-known technique to train the series data, namely image processing, video capture, and word prediction that could remember the series element using a memory cell. The main problem of handling RNN is that once it is utilized for training with long step size, it cannot remember the data for a longer period since the backpropagated gradient either shrinks or grows at every time step. This makes the training weight vanish or explode. LSTM memory overcomes this problem while a standard LSTM unit consists of input, output, and forget gates that control the data into and out of the memory cell. The structure of a single LSTM cell includes the logistic sigmoid function whereas *i*, *f*, 0, and *c* represent the input gate, forget gate, output gate, and cell state, correspondingly. The input gate determines the ratio of input and has an impact on the value of the cell state [23]. The framework could resolve the exploding and vanishing gradient problems.

Figure 3 demonstrates the framework of Bi-LSTM. Bi-LSTM has both forward and backward LSTM layers. The forward layer captures the historical data of order while the backward layer captures the future data of the sequences. The combined layers are linked to a similar resultant layer. Our network utilizes Bi-LSTM with a multihead (MH) process. MH permits the model for combined data to appear in various representations of subspaces at distinct places. The attention process plays a vital role in the DL network to capture the explicit and latent context. MH attention process is presented since it utilizes several individual attention functions to capture distinct contexts. The attention function gets input as an order of query *Q*={*Q*_1_,…, *Q*_*N*_} and group of key-value pairs {*K*, *V*}={(*K*_1_, *V*_1_),…, (*K*_*R*_, *V*_*R*_)}. MH attention method primary transforms *Q*, *K*, and *V* to *C* subspaces, with distinct and learnable linear projection.

At this point. *Q*^*c*^, *K*^*c*^, and *V*^*c*^ signify the *c*^th^ head of query, key, and value correspondingly. {*W*_*c*_^*Q*^, *W*_*c*_^*K*^, *W*_*c*_^*V*^} ∈ *ℝ*^*d*×*d*_*k*_^ implies the parameter matrices, and *d* and *d*_*k*_ stand for models and their subspace dimensions. Moreover, *C* attention functions are executed concurrently to obtain the resultant state, *O*^1^,…, *O*^*C*^.

(13) $$\begin{array}{c} O^{c}=A^{c}V^{c}\text{,}\\ A^{c}=softmax\left(\frac{Q^{c}K^{c^{T}}}{\sqrt{d_{k}}}\right)\text{.} \end{array}$$

*A* ^*c*^ implies the attention distribution, formed by *c*^th^ attention head. These resultant states are concatenated to produce the last state.

#### 3.2.4. Parameter Tuning Using WSSA Technique

In order to fine-tune the parameters involved in the DL model, the WSSA technique is used which in turn improves the classifier results. The SSA approach is stimulated from navigation behaviour of salps in search of food in the ocean [24]. It is classified as leader and follower. In the searching method of optimization technique, it is important to balance the exploration and exploitation capabilities to accomplish better efficiency. The idea of inertia weight factor is initially presented to quicken the convergence speed. Researchers find that when inertia weight is lesser, the particle has stronger exploitation capability. However, it easily falls into local optima. In contrast, when inertia weight is larger, the particle still has a stronger exploration ability; however, the searching efficacy becomes low. Furthermore, the researcher presented the inertia weight factor to enhance the searching method. Here, the weight factor reduces linearly to balance between exploration and exploitation ability; thus, the particle has a stronger global searching capability in the earlier stage and searches for the precise outcome in the later stage. In the current study, to enhance the outcomes from traditional SSA, a weight factor is included to update the position. It changes dynamically with the number of iterations [25]. The weighted factor decreases linearly with the number of iterations from maximum to minimum values to accomplish optimal outcomes.

(14) $$\begin{array}{c} w\left(t\right)=wmaX-\left(\frac{{\left(w\;\max\;-w\;\min\right)}^{⋆}t}{L}\right)\text{,} \end{array}$$

whereas *w* max and *w* min denote the maximal and minimal values of the weighted factors, *t* represents the present iteration, and *L* indicates the maximal iteration. The position is upgraded in WSSA for leader and follower and is modelled as follows:

(15) $$\begin{array}{c} X^{1}=\left\{\begin{array}{c} w^{⋆}F+c_{1}\left(\left(UB-LB\right)*c_{2}+LB\right)c_{3}\geq 0,\\ w^{⋆}F-c_{1}\left(\left(UB-LB\right)⋆c_{2}+LB\right)c_{3}\geq 0, \end{array}\right.\\ X^{j}=0.5*w*\left(X^{j}+X^{j-1}\right)\text{,} \end{array}$$

whereas the variable has a similar meaning as in SSA.

WSSA approach derives a fitness function to accomplish better classification accuracy. It describes a positive integer to characterize the improved accuracy of the candidate solution. Here, the minimization of the classification error rate is taken into account as the fitness function. The optimum solution has the least error rate whereas the worst solution achieves an increased error rate.

(16) $$\begin{array}{c} fitness\left(x_{i}\right)=classifier\;error\;rate\left(x_{i}\right)\\ =\frac{number\;of\;misclassified\;instances}{Total\;number\;of\;instances}*100\text{.} \end{array}$$

## 4. Experimental Validation

In this section, the proposed IEA-TEODL model is experimentally validated for its performance using a heart disease dataset [26]. It comprises of 270 samples with 13 attributes such as age, sex, chest pain value, resting blood sugar, serum cholesterol, fasting blood sugar, resting electrocardiographic results, maximum heart rate achieved, exercise-induced angina, old peak, slope of peak exercise, number of major vessels, and thal. Besides, the dataset includes two class labels, namely the presence of CKD and the absence of CKD.

### 4.1. Results Analysis

Table 1 and Figure 4 provide the overall results of the analysis of the IEA-TEODL model on the heart disease dataset under three runs. The results demonstrate that the proposed IEA-TEODL model accomplished an effectual classification outcome under all runs. For instance, with run-1, the IEA-TEODL model achieved a sen*s*_*y*_ of 98.76%, spe*c*_*y*_ of 93.09%, acc*u*_*y*_ of 91.27%, and an *F*_score_ of 95.61%. Along with that, with run-2, the proposed IEA-TEODL approach accomplished a sen*s*_*y*_ of 98.21%, spe*c*_*y*_ of 92.56%, acc*u*_*y*_ of 94.19%, and an *F*_score_ of 94.16%. In line with these, with run-3, IEA-TEODL methodology offered a sen*s*_*y*_ of 99.15%, spe*c*_*y*_ of 96.32%, acc*u*_*y*_ of 95.92%, and an *F*_score_ of 99.33%.

Figure 5 depicts the ROC curve generated by the IEA-TEODL approach under three runs. The figure exposes that the proposed IAOA-DLFD technique reached an enhanced outcome with maximum output under different runs. For the sample, with run-1, the proposed IEA-TEODL methodology obtained a high ROC of 97.0602. Likewise, with run-2, the IEA-TEODL algorithm obtained an enhanced outcome (ROC) of 97.4922. Eventually, with run-3, the proposed IEA-TEODL system achieved an increased ROC of 98.4221.

Figure 6 provides the accuracy and loss graph analysis results accomplished by the IEA-TEODL approach under three runs. The outcomes show that the accuracy value increased while the loss value decreased with an increase in epoch count. It can be also understood that the training loss is low, and validation accuracy is high under three runs.

### 4.2. Discussion

A brief sen*s*_*y*_ analysis was conducted on the IEA-TEODL model against existing ones, and the results are shown in Table 2 and Figure 7. The results report that the proposed IEA-TEODL model achieved better outcomes in terms of sen*s*_*y*_ under distinct instances. For instance, with 2000 instances, IEA-TEODL model reached an increased sen*s*_*y*_ of 96.58%, but NN approach, NB methodology, SVM system, and ANN models obtained reduced sen*s*_*y*_ values such as 93.55%, 87.97%, 83.16%, and 95.33% correspondingly. In addition, with 10000 instances, the proposed IEA-TEODL model reached an increased sen of 99.15%, while NN approach, NB methodology, SVM system, and ANN models obtained reduced sen*s*_*y*_ values such as 93.47%, 88.26%, 84.21%, and 98.70%, respectively.

A comparative spe*c*_*y*_ analysis was conducted on the IEA-TEODL model against existing ones, and the results are shown in Table 3 and Figure 8. The results report that the proposed IEA-TEODL approach achieved better outcomes in terms of spe*c*_*y*_ under various instances. For instance, with 2000 instances, IEA-TEODL approach reached an increased spe*c*_*y*_ of 95.40%, whereas NN approach, NB methodology, SVM system, and ANN models obtained the least spe*c*_*y*_ values such as 84.86%, 83.71%, 80.93%, and 94.36% respectively. Furthermore, with 10000 instances, the proposed IEA-TEODL technique reached an increased spe*c*_*y*_ of 96.32%, whereas NN approach, NB methodology, SVM system, and ANN methodologies obtained less spe*c*_*y*_ values such as 90.26%, 86.91%, 84.13%, and 91.90% correspondingly.

A detailed acc_*y*_ analysis was conducted on the IEA-TEODL algorithm against existing methods, and the results are shown in Table 4 and Figure 9. The results report that the proposed IEA-TEODL technique achieved better outcomes with respect to acc_*y*_ under distinct instances. For instance, with 2000 instances, the proposed IEA-TEODL model attained an increased acc_*y*_ of 94.28%, but NN approach, NB methodology, SVM system, and ANN systems obtained less acc_*y*_ values such as 88.73%, 77.43%, 73.17%, and 92.54% correspondingly.

Additionally, with 10000 instances, the proposed IEA-TEODL approach reached the maximum acc_*y*_ of 95.92%, whereas NN approach, NB methodology, SVM system, and ANN models obtained low acc_*y*_ values, namely 89.61%, 82.02%, 81.98%, and 93.88% correspondingly.

A brief *F*_score_ analysis was conducted between the IEA-TEODL method and the existing models, and the results are shown in Table 5 and Figure 10. The results infer that the proposed IEA-TEODL approach achieved better outcomes in terms of *F*_score_ under distinct instances. For instance, with 2000 instances, the presented IEA-TEODL model reached the maximum *F*_score_ of 98.32%, while NN approach, NB methodology, SVM system, and ANN algorithms obtained low *F*_score_ values such as 92.33%, 84.63%, 81.59%, and 97.67% correspondingly. Finally, with 10000 instances, the proposed IEA-TEODL algorithm obtained an increased *F*_score_ of 99.33%, whereas NN approach, NB methodology, SVM system, and ANN models reached less *F*_score_ values such as 97.71%, 84.25%, 82.32%, and 95.84% correspondingly.

At last, a brief TEC examination was conducted between IEA-TEODL model and recent methods, and the results are shown in Table 6 and Figure 11 [27]. The experimental values highlight that the proposed IEA-TEODL model produced effective TEC values under distinct IoT sensor counts. For instance, with 100 IoT sensors, the IEA-TEODL model gained a low TEC of 41.30%, whereas EE-PSO, ABC, GWO, and ACO algorithms obtained high TEC values such as 45.04%, 57.14%, 60.65%, and 66.16%, respectively. At the same time, with 300 IoT sensors, the proposed IEA-TEODL method gained a low TEC of 57.71%, whereas EE-PSO, ABC, GWO, and ACO systems obtained high TEC values such as 59.73%, 67.24%, 73.44%, and 77.15% correspondingly. In line with this, with 500 IoT sensors, the proposed IEA-TEODL model gained a low TEC of 65.74%, whereas EE-PSO, ABC, GWO, and ACO approaches attained high TEC values namely 69.28%, 78.51%, 82.11%, and 84.08% correspondingly.

After examining the above-mentioned tables and figures, it is apparent that the proposed IEA-TEODL technique outperformed other methods. The enhanced performance of the proposed model is due to the integration of EACTEO-C-based cluster construction and optimal DL-based disease classification.

## 5. Conclusion

In this study, a novel IEA-TEODL technique has been developed to accomplish clustering and decision-making in an IoT-enabled smart healthcare environment. The proposed IEA-TEODL technique follows a two-stage process, namely EACTEO-C-based cluster construction and optimal DL-based disease classification. Besides, the disease diagnosis model encompasses a series of subprocesses, namely preprocessing outlier removal, MHA-BLSTM-based classification, and WSSA-based hyperparameter optimization. In order to validate the promising performance of the proposed IEA-TEODL technique, a wide range of simulations was conducted against benchmark datasets. The simulation results established the enhanced outcomes of the IEA-TEODL technique over other recent techniques under distinct evaluation metrics. Thus, the IEA-TEDOL technique can be utilized as an effectual tool to accomplish energy efficiency and data classification in an IoT environment. In the future, lightweight cryptography and authentication mechanisms can be included to assure security in the smart healthcare environment.

## Figures and Tables

**Figure 1:** Smart healthcare systems [4].

**Figure 2:** Block diagram of IEA-TEODL technique.

**Figure 3:** Bi-LSTM structure [23].

**Figure 4:** Analytical results of IEA-TEODL technique under three runs.

**Figure 5:** ROC analysis results of IEA-TEODL technique under three runs.

**Figure 6:** Accuracy and loss analysis results of IEA-TEODL technique under three runs.

**Figure 7:** sen*s*_*y*_ analysis of the IEA-TEODL technique with recent approaches.

**Figure 8:** Spe*c*_*y*_ analysis results of the IEA-TEODL technique against recent approaches.

**Figure 9:** Acc_*y*_ analysis results of the IEA-TEODL technique against recent approaches.

**Figure 10:** *F*_score_ analysis results of the IEA-TEODL technique against recent approaches.

**Figure 11:** TEC analysis of IEA-TEODL technique with recent approaches.

**Table 1:** Analytical results of IEA-TEODL technique under three runs.

No. of runs	Sensitivity	Specificity	Accuracy	*F*-score
Run-1	98.76	93.09	91.27	95.61
Run-2	98.21	92.56	94.19	94.16
Run-3	99.15	96.32	95.92	99.33
Average	98.71	93.99	93.79	96.37

**Table 2:** Sensitivity analysis results of IEA-TEODL technique against existing approaches.

Instances	Nearest neighbour	Naive Bayes	SVM model	ANN model	IEA-TEODL
2000	93.55	87.97	83.16	95.33	96.58
4000	88.03	85.03	81.95	94.33	95.41
6000	92.92	86.87	83.62	95.53	97.41
8000	92.02	88.98	81.40	96.96	98.71
10000	93.47	88.26	84.21	98.70	99.15

**Table 3:** Specificity analysis results of IEA-TEODL technique against existing approaches.

Instances	Nearest neighbour	Naive Bayes	SVM model	ANN model	IEA-TEODL
2000	84.86	83.71	80.93	94.36	95.40
4000	86.58	84.08	82.75	92.92	95.29
6000	86.72	86.59	84.01	94.27	96.14
8000	87.65	81.34	78.14	92.26	94.40
10000	90.26	86.91	84.13	91.90	96.32

**Table 4:** Accuracy analysis results of the IEA-TEODL technique against existing approaches.

Instances	Nearest neighbour	Naive Bayes	SVM model	ANN model	IEA-TEODL
2000	88.73	77.43	73.17	92.54	94.28
4000	90.97	77.80	76.69	94.33	95.86
6000	86.99	76.89	75.86	92.59	93.70
8000	86.43	80.42	77.86	94.82	95.15
10000	89.61	82.02	81.98	93.88	95.92

**Table 5:** *F*-score analysis results of the IEA-TEODL technique against existing approaches.

Instances	Nearest neighbour	Naive Bayes	SVM model	ANN model	IEA-TEODL
2000	92.33	84.63	81.59	97.67	98.32
4000	89.47	84.91	82.45	95.87	96.87
6000	92.57	88.19	87.16	95.33	96.52
8000	92.28	83.73	80.61	94.49	96.29
10000	91.71	84.25	82.32	95.84	99.33

**Table 6:** Results of the analysis of total energy consumption (%) between the existing and the proposed methods.

IoT sensors	IEA-TEODL	EE-PSO model	ABC model	GWO model	ACO model
100	41.30	45.04	57.14	60.65	66.16
200	49.85	52.35	61.01	68.66	74.26
300	57.71	59.73	67.24	73.44	77.15
400	60.99	63.72	72.49	76.00	81.06
500	65.74	69.28	78.51	82.11	84.08

## Data Availability

Data sharing is not applicable to this article as no datasets were generated during the current study.
